The article "Developing a Recognition System for Diagnosing Melanoma Skin Lesions Using Artificial Intelligence Algorithms" was published in 2021. Journal: Comput Math Methods Med.

# Developing a Recognition System for Diagnosing Melanoma Skin Lesions Using Artificial Intelligence Algorithms

**DOI:** 10.1155/2021/9998379

**Published:** 2021-05-15

**Authors:** Fawaz Waselallah Alsaade, Theyazn H. H. Aldhyani, Mosleh Hmoud Al-Adhaileh

**Affiliations:** ^1^College of Computer Science and Information Technology, King Faisal University, P.O. Box 400, Al-Ahsa, Saudi Arabia; ^2^Community College of Abqaiq, King Faisal University, P.O. Box 400, Al-Ahsa, Saudi Arabia; ^3^Deanship of E-Learning and Distance Education, King Faisal University, Saudi Arabia, P.O. Box 400, Al-Ahsa, Saudi Arabia

## Abstract

In recent years, computerized biomedical imaging and analysis have become extremely promising, more interesting, and highly beneficial. They provide remarkable information in the diagnoses of skin lesions. There have been developments in modern diagnostic systems that can help detect melanoma in its early stages to save the lives of many people. There is also a significant growth in the design of computer-aided diagnosis (CAD) systems using advanced artificial intelligence. The purpose of the present research is to develop a system to diagnose skin cancer, one that will lead to a high level of detection of the skin cancer. The proposed system was developed using deep learning and traditional artificial intelligence machine learning algorithms. The dermoscopy images were collected from the PH2 and ISIC 2018 in order to examine the diagnose system. The developed system is divided into feature-based and deep leaning. The feature-based system was developed based on feature-extracting methods. In order to segment the lesion from dermoscopy images, the active contour method was proposed. These skin lesions were processed using hybrid feature extractions, namely, the Local Binary Pattern (LBP) and Gray Level Co-occurrence Matrix (GLCM) methods to extract the texture features. The obtained features were then processed using the artificial neural network (ANNs) algorithm. In the second system, the convolutional neural network (CNNs) algorithm was applied for the efficient classification of skin diseases; the CNNs were pretrained using large AlexNet and ResNet50 transfer learning models. The experimental results show that the proposed method outperformed the state-of-art methods for HP2 and ISIC 2018 datasets. Standard evaluation metrics like accuracy, specificity, sensitivity, precision, recall, and *F*-score were employed to evaluate the results of the two proposed systems. The ANN model achieved the highest accuracy for PH2 (97.50%) and ISIC 2018 (98.35%) compared with the CNN model. The evaluation and comparison, proposed systems for classification and detection of melanoma are presented.

The article "Developing a Recognition System for Diagnosing Melanoma Skin Lesions Using Artificial Intelligence Algorithms" was published in 2021. Journal: Comput Math Methods Med.

## 1. Introduction

Skin is the largest organ of the human body. It protects the body's internal tissues from the external environment. The skin also helps maintain the body temperature at a steady level and shields our body from unfortunate solar radiation, for example, bright (UV) light introduction. It counteracts contaminants and permits the generation of vitamin D and is essential for certain body capacities [1]. Melanoma is an abnormal proliferation of skin cells that arises and develops, in most cases, on the surface of the skin that is exposed to copious amounts of sunlight. However, this common type of cancer can also develop in areas of the skin that is not exposed to too much sunlight.

Melanoma is the fifth most common lesion of skin cancer. As recently reported by the Skin Cancer Foundation (SCF), it is considered the most serious form of skin cancer because it is capable of spreading to other parts of the body. Once melanoma spreads elsewhere, it becomes difficult to treat. However, early detection protects lives, that is rare but the most dangerous. In the past couple of years, the incidence of skin cancer has been increasing, and reports show that the recurrence of melanoma occurs at regular intervals [2]. Skin disease, the most overwhelming kind of malignancy, manifests when skin cells lose control. There are three primary kinds of skin growths: basal cell skin tumors (basal cell carcinomas), squamous cell skin malignancies (squamous cell carcinomas), and melanomas. For the most part, skin growths that are not melanomas are normally grouped into nonmelanoma skin tumors. Skin cancer disease can be classified into two groups: benign and malignant. Benign cancers are classified as basal cell carcinoma and squamous cell carcinoma. Malignant cancer (aka melanoma) is the most dangerous and leads to death. Skin tumors are the costliest malignancies [3].

The National Cancer Institute (NCI) has reported that melanoma is one of the most serious types of cancers. When too many ultraviolet (UV) lights hit the skin, over time, it leads to DNA damage in skin cells, causes cancer and takes many years. Cancerous melanoma is one of the fastest rising skin cancer in the world, with more than 70,000 projected new cases in the USA alone and an estimated 10,000+ deaths just in 2017, according to the American Cancer Society (ACS) [4]. In 2012, around three million skin lesions were evaluated in the US, and over 100,000 were diagnosed as malignant melanoma [5].

Artificial intelligence (AI) algorithms have advanced at a notable rate and have found practical applications in various industries [6]. AI algorithms define training data inputs to training data outputs by designing a complex structure of layers for solving specific problems. Currently, deep learning algorithms are employed to solve problems that are barely resolvable via traditional ANNs [7]. ANNs were applied to large amounts numbers of scientific data, learning from complex data [8, 9], developing recognition systems using image processing [10], used them for analysis and classification of texts [11], etc. One of the important applications of ANNs is for biomedical diagnosis [12, 13]. In addition, ANNs were used to analyze health informatics [14] using biomedical data [15] and magnetic resonance imaging (MRI) as the diagnostic system [16]. The artificial intelligence algorithms were applied to achieve numerous biomedical tasks, such as a biomedical segmentation image to determine the specific disease areas, develop diagnostic systems, classify all types of diseases, predict diseases using health informatics, and detect various anatomical regions of interest (ROI). Currently, the deep learning algorithms were successfully developed superior biomedical health.

The article "Developing a Recognition System for Diagnosing Melanoma Skin Lesions Using Artificial Intelligence Algorithms" was published in 2021. Journal: Comput Math Methods Med.

In recent years, several researchers were applied to various AI algorithms to diagnose skin cancer. Different dermatological datasets were used to test their proposed research models. Zhou developed a diagnostic system using several mean shift-based techniques for segmenting skin lesions during the acquisition of dermatoscopic images [17–19]. Garnavi et al. applied optimal color channels and hybrid thresholding algorithms in order to segment skin lesions [20]. In more recent research, Pennisi et al. presented Delaunay triangulation (DT) to divide skin lesion regions into segments [21]. Ma et al. [22] presented a novel defined speed function and stopping approach for the segmentation of skin lesions. The method is more robust against noise and proves effective and flexible at segmenting skin lesions. Yu et al. [23] proposed a fully convolutional residual network (FCRN) for skin lesion segmentation. Celebi et al. applied an extraction method to obtain features, including color and texture, as well as process these features using classification algorithms [24]. Schaefer applied an automatic border detection technique to segment the skin lesion area and extract features, such as shape, texture, and color, for the diagnosis of melanoma [25, 26]. Codella et al. developed hybrid CNNs and support vector machines (SVMs) to detect melanoma [27]. Wichakam et al. utilized CNNs to extract features for melanoma in order to design a recognition system [28].

The main contribution of the proposed research can be summarized as follows: the key to deep learning capabilities lies in the of the neural networks' ability to learn from data through generally purpose learning procedures. The proposed research addresses the application of AI in the medical diagnosis of skin diseases. The main challenges in our work were how to differentiate between benign and malignant images.  Figure 1 illustrates skin cancer samples from diverse datasets.

The article "Developing a Recognition System for Diagnosing Melanoma Skin Lesions Using Artificial Intelligence Algorithms" was published in 2021. Journal: Comput Math Methods Med.

The early detection of melanoma and improving dermatologic techniques can increase family physicians' confidence in their referral accuracy to dermatologists, thereby, decreasing unnecessary surgery or biopsies (excisions). Early detection could reduce mortality and increase the survival rate of patients with melanoma to 98%. These are the main purposes of our research. A comparative analysis of performance between artificial neural networks (ANNs) and convolution neural networks (CNNs) are presented along with the research of simple, suitable segmentation techniques for obtaining ROI. These techniques were applied to two dermoscopy dataset images, namely, PH2and ISIC 2018, using different feature extraction methods to obtain diagnostic accuracy in the early detection of melanoma.

## 2. Materials and Methods

Since the nature of characteristics of each dataset is different, and the challenges in each dataset are different too; these challenges composed of lesion segmentation, disease classification and detection, localization of visual dermoscopy features/pattern, and lesion attribute detection. Due to this reason, the proposed system has the ability detection of melanomas in dermoscopy images.  Figure 2 displays the framework of the proposed system for the classification of skin diseases. In feature-based, the active count segmentation algorithm was used to segment ROI from dermoscopy images. The hybrid features extraction local binary pattern and Gray Level Co-occurrence Matrix (GLCM) methods to extract texture features. These features were processed by an artificial neural network algorithm. The second system, convolutional neural networks (CNNs), was applied for efficient classification of skin disease; the CNNs were pretrained using large AlexNet and ResNet50 methods. This work is aimed at determining the best selected of a system for skin lesion classification. The other objective is to compare the robust and reliability between the deep leaning and traditional ANN algorithms.

### 2.1. Datasets

In this present research work, two real standard datasets, namely, PH2 and ISIC2018, were used to develop a recognition system for detecting skin diseases.

#### 2.1.1. PH2 Dataset

The PH2 dataset is real dermoscopy images; it was used to evaluate performances of the proposed system for the classification of skin diseases. In studies, 120 dermoscopy images were considered, and it is divided into 40 atypical nevi, 40 melanoma, and 40 common nevus. The total equaled 120 dermoscopy images; Figure 3 shows the sample of the PH2 dataset. The PH2 dermoscopy images are JPG format. The resolution of the images is 766 × 560: https://www.fc.up.pt/addi/ph2%20database.html.

The article "Developing a Recognition System for Diagnosing Melanoma Skin Lesions Using Artificial Intelligence Algorithms" was published in 2021. Journal: Comput Math Methods Med.

#### 2.1.2. ISIC 2018 Dataset

In order to simulate and evaluate the proposed method, the ISIC 2018 dataset was used. The ISIC 2018 stands for the International Skin Imaging Collaboration. It contains a large number of lesion diagnosed images through their ISIC 2018 project. The archive of ISIC is presented by three large databases, such as BCN_20000, HAM 10000, and MSK. The HAM dataset has seven classes, namely, melanocytic nevi (nv) 200, melanoma (mel) 200, benign keratosis lesions (bkl) 200, basal cell carcinoma (bcc) 22, actinic keratoses (akiec) 22, vascular (vasc) 100, and dermatofibroma (df) 100.  Figure 4 shows the sample from the ISIC 2018 dataset with different skin diseases: https://dataverse.harvard.edu/dataset.xhtml?persistentId=doi:10.7910/DVN/DBW86T.

### 2.2. Preprocessing Stages

In this section, the preprocessing steps were applied to obtained significant features from dermoscopy images.  Figure 5 shows the preprocessing stages of the proposed methodology.

#### 2.2.1. Gaussian Filter Method

A Gaussian filter method is used to apply a 2-D convolution operator to “blur” the skin images and remove details and noise. It uses the kernel function for representing the shape of a Gaussian. The function is defined as the following:

(1) $$\begin{array}{c} \;h\left(x,y\right)=\frac{1}{2\pi \;\sigma^{2}}\text{e}\frac{x^{2}-y^{2}}{2\sigma^{2}}, \end{array}$$

where *σ* is the standard deviation parameter of the distribution.

#### 2.2.2. Segmentation Method

The snake model is one of the active contour types; it has the ability to perform appropriate segmentation. The model clearly identifies the target lesion and requires prior knowledge about the contour of the particular lesion or complex lesion. The active snake model applies spline, which focuses on the minimum energy followed by different forces that control the image. The spline A mathematical function of a polynomial set to derive geometric figures and curves in the image. Geometric active contours are applied by [29, 30].

The curve ∁ is represented in by a level set function∅: *Ω* ⟶, where is zero at the border region in the image of skin lesions *I*. The curve ∁ divides the subregions *W*_*k*_⊂*Ω* into two subregions *w*, *w*, with *ϕ*, where

(2) $$\begin{array}{c} \text{inside}\left(∁\right)=w=\left\{x\in w_{k}:\emptyset \left(x\right)>0\right\},\\ \text{outside}\left(∁\right)=w=\left\{x\in \Omega :\emptyset \left(x\right)<0\cup x\in \Omega \backslash w_{k}\right\}. \end{array}$$

In this algorithm, the level set evolution starts by moving contour inwards. The initial contour is determined at the boundaries of the image in order to calculate the contour map of the skin lesion area. When *ϕ* > 0 is set, the level set moves inward, to compute the subregion of the zero levels. The outer region is also computed by subtracting the previously subregion computed subregion from the current region computed, as shown by the equations below.

(3) $$\begin{array}{c} w_{0}=w_{1}+{\bar{w}}_{1}\Rightarrow {\bar{w}}_{1}=w_{0}-w_{1},\\ {\bar{w}}_{2}={\text{w}}_{1}-{\text{w}}_{2},\\ {\bar{w}}_{3}={\text{w}}_{2}-{\text{w}}_{3}. \end{array}$$

On the whole, the outer subregion can be computed as

(4) $$\begin{array}{c} {\bar{w}}_{\text{k}}={\text{w}}_{\text{k}-1}–{\text{w}}_{\text{k}}. \end{array}$$

When segmentation, the active contour algorithm moves dynamically towards the boundaries of the object. In order to achieve this, external energy moves the zero level towards the boundaries of the object. The following equation illustrates the energy functional for the function 𝜙.

(5) $$\begin{array}{c} w_{spf}\left(\emptyset \right)=\lambda L_{spf}\left(\emptyset \right)+\nu \;A_{spf}\left(\emptyset \right)\; \end{array}$$

where *λ* > 0 and *ν* are constants. The terms *L*_*spf*_ and *A*_*spf*_ are defined in the following equations

(6) $$\begin{array}{c} L_{\text{spf}}\left(\emptyset \right)=\int_{\Omega }\text{spf}\left(I\right)\delta_{\varepsilon }\left(\emptyset \right)\left|\nabla \emptyset \right|dx,\\ A_{\text{spf}}\left(\emptyset \right)=\int_{\Omega }\text{spf}\left(I\right)H_{\varepsilon }\left(\emptyset \right)\left(-\emptyset \right)dx, \end{array}$$

where spf (*I*) will be defined later in the equation (), *H*_*ε*_ is the Heaviside function, and *δ*_*ε*_ denotes the univariate Dirac delta function that will be defined later. 𝐿spf (𝜙) is reduced by driven the zero-level curve *C* into a smooth curve, so that small energy in spf (*I*) speeds up curve evolution, which will drive the zero level set toward the boundaries of a skin lesion. The coefficient *v* of *A*_spf_ (*ϕ*) is a positive or negative value according to the position of the initial contour of the region of interest. If the initial contour is outside the region of interest, then the value of *v* is positive, and if its position is inside the region of interest, then the value of *v* is negative in order to speed up the expansion of contours.

The article "Developing a Recognition System for Diagnosing Melanoma Skin Lesions Using Artificial Intelligence Algorithms" was published in 2021. Journal: Comput Math Methods Med.

We define a new region according to energy functional. We suggest the *E*_proposed_ for the previously used SPF function. Let *I* : *Ω*⟶*R* be the image of the inputted skin lesion and *C* be a closed curve, and the energy functional proposed is defined as follows.

(7) $$\begin{array}{c} E_{\text{proposed}}=\int_{\Omega }{\left|\text{I}\left(\text{x}\right)-C_{1}\right|}^{2}H_{\varepsilon }\left(\emptyset \left(x\right)\right)M^{k}\left(x\right)dx+\int_{\Omega }{\left|\text{I}\left(\text{x}\right)-C_{1}\right|}^{2}\left(1-H_{\varepsilon }\left(\emptyset \left(x\right)\right)\right)M^{k}\left(x\right)dx. \end{array}$$

Keeping 𝜙 constant while reducing energy *E* proposed by the following formulas, we get *C*_1_ for the *w* region and *C*_1_ for the $\bar{w}$ region as follows.

(8) $$\begin{array}{c} C_{1}\left(\phi \right)=\frac{\int_{\Omega }\;I\left(x\right)\;H_{\varepsilon }\left(\emptyset \left(x\right)\right)M^{k}\left(x\right)dx}{\int_{\Omega }H_{\varepsilon }\left(\emptyset \left(x\right)\right)M^{k}\left(x\right)dx},\\ C_{2}\left(\phi \right)=\frac{\int_{\Omega }I\left(x\right)\left(1-H_{\varepsilon }\left(\emptyset \left(x\right)\right)\right)M^{k}\left(x\right)dx}{\int_{\Omega }\left(1-H_{\varepsilon }\left(\emptyset \left(x\right)\right)\right)M^{k}\left(x\right)dx}. \end{array}$$

*M* ^*k*^ is the characteristic function of the defined subregion as follows:

(9) $$\begin{array}{c} M^{k}\left(x\right)=\phi >0,\\ M^{0}:\Omega ⟶-1. \end{array}$$

By calculating of variations *A*_sp*f*_(∅), it can be written as the Gateaux derivative (first variation) as follows:

(10) $$\begin{array}{c} Q\left(\emptyset \right)=\left(\lambda .\mathrm{div}\left(\text{spf}\left(I\right).\frac{\nabla \emptyset }{\left|\nabla \emptyset \right|}\right)+\nu .\text{spf}\left(I\right)\right)\delta_{\varepsilon }\left(\emptyset \right). \end{array}$$

A function 𝜙 which minimizes the function and satisfies the Euler Lagrange function as with the equation *∂E*_spf_/*∂*∅ = 0. The first term corresponds to *L*_spf_, which indicates the object's curvature according to the edges' information, while the second term corresponds to *A*_spf_, which indicates a region within the region of interest. If the value of SPF is positive, then the contour moves to the region of high density and vice versa.

An iterative process to minimize the function *E*_spf_ (*ϕ*) through gradient flow with time *t* by the following formula:

(11) $$\begin{array}{c} \phi_{\left(t=0\right)}=\phi_{0},\frac{\partial \emptyset }{\partial t}=Q\left(\emptyset \right). \end{array}$$

An SPF function is a mathematical expression with two values in the range [1, -1] inside and outside the region of interest. There are many ways to calculate the SPF function, some of them have global density, and some have a local density in their construction. We proposed a new SPF function restricted to the term mask that works to evolution the level set into inwards. When the mask is set to 1, it modifies the compressive force signals so that when it is outside the object, the contour shrinks, and when it is inside the object, the contour expands.

The article "Developing a Recognition System for Diagnosing Melanoma Skin Lesions Using Artificial Intelligence Algorithms" was published in 2021. Journal: Comput Math Methods Med.

The global fitted model for a level set function defined as follows:

(12) $$\begin{array}{c} I_{\text{GFI}}=c_{1}H_{\varepsilon }\left(\emptyset \right)+c_{1}\left(1-H_{\varepsilon }\left(\emptyset \right)\right), \end{array}$$

According to the global fitted model mentioned above, the SPF function is reformulated as follows:

(13) $$\begin{array}{c} \text{spf}\left(I\right)=\left\{\begin{array}{c} \;\frac{\left(\text{I}\left(x\right)-I_{\text{GFI}}\right)\;M^{k}}{\max\left(\left|\text{I}\left(x\right)-I_{\text{GFI}}\right|\right)}I\left(x\right)\neq 0,\\ 0\;I\left(x\right)=0. \end{array}\right. \end{array}$$

In this work, the Dirac function *δ*_*ε*_(*z*) and Heaviside function *H*_*ε*_(*z*) are the smoothed versions of the whole image. The approximation for *H*_*ε*_(*z*) and *δ*_*ε*_(*z*) is as follows:

(14) $$\begin{array}{c} {\text{H}}_{\varepsilon }\left(z\right)=\frac{1}{2}\left(1+\frac{2}{\pi }\arctan\left(\frac{z}{\varepsilon }\right)\right),\\ \delta_{\varepsilon }\left(z\right)=\frac{\varepsilon }{\pi \;\left(z^{2}+\varepsilon^{2}\right)}. \end{array}$$

If there is a difference between the initial level set function and SDF, then schema reinitialization is unable to reinitialization SDF. In our proposed, the initial level 𝜙_0_ is set as in the formula.

(15) $$\begin{array}{c} \phi \left(\text{x},\text{t}=0\right)=\left\{\begin{array}{c} -\rho \;x\in \Omega_{0}-\partial \Omega_{0}\\ 0x\in \partial \Omega_{0}\\ \rho x\in \Omega -\Omega_{0} \end{array},\right. \end{array}$$

where *ρ* > 0 is a constant value and 𝜙0 with *ρ* = 2 that is used.

When the pixels are similar between two consecutive contours, the contour algorithm will stop using the stop value at a certain point.

If

(16) $$\begin{array}{c} \;\overset{\text{row}}{\underset{i=0}{\sum }}\overset{\text{col}}{\underset{j=0}{\sum }}M_{i,j}^{k}<\left(\frac{\text{stopping value}}{100}\right)\overset{\text{row}}{\underset{i=0}{\sum }}\overset{\text{col}}{\underset{j=0}{\sum }}\text{o}\text{ld}M_{i,j}^{k}, \end{array}$$

then the contour will stop moving.

*ldM*_*i*,*j*_^*k*^ denotes the last calculated mask for the contour, and *M*_*i*,*j*_^*k*^ indicates to the current mask of the contour; row and col are the maximum number of rows and columns, respectively, in the skin lesion images. The stop value is in a range between 98 and 100, which is calculated by computing the mean intensity value in the initial contour. The threshold value *T* is used to eliminate small values when calculating the stop value. The active contour method was developed to extract the region of interest (ROI) from dermoscopy images. It is noted that the active contour method was appropriate for dermoscopy images.  Figure 6 displays the region of interests of PH2, whereas the important region of skin lesions for ISIC 2018 dermoscopy images is presented in Figure 7.

The article "Developing a Recognition System for Diagnosing Melanoma Skin Lesions Using Artificial Intelligence Algorithms" was published in 2021. Journal: Comput Math Methods Med.

### 2.3. Feature Extraction

In this present research, we fused two feature extractions: the Local Binary Pattern (LBP) and GLCM method to extract features from the dermoscopy images [31]. The Local Binary Pattern (LBP) is one of the important features of the extraction method; it has implemented many image processing fields. The local binary pattern method was proposed by Ojola [32], to extract the significant texture feature from the pixel values. The LBP is a very simple and robust method for extracting in each center pixel of the input image (*x*, *y*) with grey level values of the *ℊ*_*c*_, and the LBP method is computed by comparing the *ℊ*_*c*_ values of grey pixels at the *R* distance during its *P* neighborhood pixels.  Figure 8 shows the LBP neighborhood pixels, either clockwise or counterclockwise. (*x*, *y*) has grey level values than neighborhood *p* that will assign 0 or 1 values.  Figure 8 displays a sample 2D plot of the LBP method for extracting the features from the ROI that has obtained by the segmentation method.

Its LBP value is estimated by comparing the *g*_*c*_ value with the grey level values of pixels at the *R* distance within its surrounding *P* neighborhood pixels following the pixels along a circular path either clockwise or counterclockwise. The LBPP, *R*, is computing as follows:

(17) $$\begin{array}{c} {\text{LBP}}^{P,R}\left(x_{c},y_{c}\right)=\overset{p-1}{\underset{p=0}{\sum }}s{\left(g_{i}^{P,R}-g_{c}\right)}^{2^{i-1}}, \end{array}$$

where *x* is defined

(18) $$\begin{array}{c} s\left(x\right)=\left\{\begin{array}{c} 1,\text{if }x\geq 0\\ 0,\text{if }x<0 \end{array}\right.. \end{array}$$

The GLCM method is one of powerful statistical extraction feature methods. The GLCM method uses to extract the texture features from dermoscopy image. We considered 13 statistical features, namely, contrast, correlation, energy, homogeneity, mean, standard deviation, entropy, RMS, variance, smoothness, kurtosis, and skewness. We fused the features of GLCM with LBP to obtain robust features. 216 significant features were selected from the hybrid method for training the classification algorithms.

The article "Developing a Recognition System for Diagnosing Melanoma Skin Lesions Using Artificial Intelligence Algorithms" was published in 2021. Journal: Comput Math Methods Med.

### 2.4. Classification Algorithms

In this section, the classification algorithm artificial neural networks (ANNs) and convolutional neural networks (CNNs) were applied to detect skin diseases from dermoscopy images.

#### 2.4.1. Artificial Neural Networks (ANNs)

The artificial neural network is a very powerful computation method for developing numbers of real medical applications. In general, the neural network (NN) models are used as a very powerful machine learning algorithms for time-series prediction of different engineering applications. The ANN model is consist of an input layer, hidden layers, and an output layer. Each hidden layer has weight and bias parameters to manage neurons. In order to transfer the data from the hidden layer into the output layer, the activation function is used. The learning algorithms are used to select the weights within the NN framework. The weight selection is based on the minimum performance measures such as mean square error (MSE).  Figure 9 shows the architecture of ANNs for detecting skin diseases.

In this study, the ANN algorithm has applied for diagnosis the skin diereses. The ANNs have three significant layers input, hidden layer, and output layers. Two standard real datasets have such as ISIC 2018 and PH2 employed to examine the proposed methodology. Two thousand sixteen features were considered input training for both datasets, whereas five hidden layers transfer the input training from input to output the sigmoid function. However, the output layer for PH2 dataset is 3 and 7 output for HAM dataset—the sigmoid function.

#### 2.4.2. Deep Learning with Convolutional Neural Networks (CNNs)

A convolutional neural network (CNNs) system is used for deep learning. In signal processing and image processing domain, such methods are commonly used to classify the scenes and objects as well as to perform the ROI detection and segmentation process [32–39]. In this work, two transfer models of CNN algorithms, namely, AlexNet and ResNet50, were applied to classify skin diseases.  Figure 10 shows the framework of the CNN algorithm. It gets rid of the process of manual feature extraction as the learning of features is directly performed by CNNs. In the convolutional layer, given the input, a weight matrix passes all over the input, and the recorded weighted summation is placed as a single element of the subsequent layer. Three hyperparameters include (filter size, stride, and zero padding) that affect the performance of the convolutional layer. By using different values for these hyperparameters, the convolutional layer will decrease the complexity of the network. The CNN algorithm has different layers.

Many nonlinear functions can be used in the convolutional neural network. However, Rectified Linear Unit ReLU is one of the most common nonlinear functions applied in image processing applications. The ReLU is shown in Figure 11. The main goal of using the ReLU is applying element-wise activation function to the feature map from the previous layer. In addition, the ReLU function transfers all value of features map to positive or zero. The ReLU can be represented, as shown in Eq. (1).

(19) $$\begin{array}{c} \text{ReLU}\left(x\right)=\left[0\;\text{if }x<0,x\;\text{if }x>=0\right]. \end{array}$$

The pooling layer, roughly, reduces the dimensions of the input data and minimizes the number of parameters in the feature map. The simplest way to implement the pooling layer is by selecting the maximum of each region and then writing it in the next layer's corresponding place. Using this pooling filter reduces the input size to 25% of its original size. Also, averaging represents another pooling method. However, taking the maximum is the most popular and promising method in the literature. The maximum pooling method is noninvertible; so, the original values before pooling operation cannot be restored. But if the locations of the maximum values of each moving in a set of switch variables are recoded, approximate original values can be generated.

The article "Developing a Recognition System for Diagnosing Melanoma Skin Lesions Using Artificial Intelligence Algorithms" was published in 2021. Journal: Comput Math Methods Med.

The softmax function is used to calculate the probability distribution of an *N*-dimensional vector. The main purpose of using softmax at the output layer is the multiclass classification method in machine learning algorithms, deep learning, and data science. The correct calculation of the output probability helps to determine the proper target class for input dataset. The probability of the maximum values is increased using the exponential element. The softmax equation is shown by Eq. (19).

(20) $$\begin{array}{c} O_{i}=\frac{e^{z_{i}}}{\sum_{i=1}^{M}e^{z_{i}}}, \end{array}$$

where *i*, *z*_*i*_, is the output, the *O*_*i*_ indicates to the softmax output, and *M* is the total number of output nodes.

The fully connected layer represents the last layers in any convolutional neural network. Each node in the layer (*L*) is connected directly to each node in layers (*L* − 1) and (*L* + 1). There is not any connection between nodes in the same layer in contrast with the traditional ANN. Therefore, this layer takes long training and testing time. More than one fully connected layer can be used at the same network, as shown in Figure 12.

In this study, two transfer learnings, namely, the AlexNet and ResNet50 models, are implemented, and the detailed description of these models is as follows:

*(1) AlexNet Model*. AlexNet contains five convolutional layers, as well as two fully connected layers for learning features. It has max-pooling after the first, second, and fifth convolutional layer. In total, it has 650 K neurons, 60 M parameters, and 630 M connections. The AlexNet was the first to show that deep learning was effective in computer vision tasks [54, 84]. Each convolutional network is made up of convolutional layer, nonlinearity, pooling layer, one fully connected layer and, lastly, softmax are considered for recognition of the gestures.  Table 1 shows the parameters of the CNN algorithm.  Figure 13 shows the proposed framework of the AlexNet transfer learning model.

*(2) ResNet50 Model*. The ResNet models, developed by He et al. [41], are a powerful transfer learning model of CNNs for classification purposes. They have good convergence behaviors and compelling accuracy. The ResNet transfer learning model was built with different layers, like 18, 34, 50, 101, 152, and 1202. These layers gave the ResNet more efficiency to obtain the best accuracy. The ResNet transfer learning model is similar to the VGG net; nonetheless, ResNet50 is eight times deeper than VGG [42]. The ResNet50 consists of 49 convolutional layers and a fully connected layer at the end of the network. Finally, the ResNet50 was applied to classify skin diseases.  Table 2 shows the significant parameters of ResNet50.

The article "Developing a Recognition System for Diagnosing Melanoma Skin Lesions Using Artificial Intelligence Algorithms" was published in 2021. Journal: Comput Math Methods Med.

There are several layers in CNNs to detect various features of input image through each layer learning. At different resolutions, filters are applied to every trained image, and the outcome of every convolved image is utilized in the next layer as input. We used the CNNs for disease detection based on extracted features from the input disease. Our aim behind using the CNNs for skin disease detection is to improve the recognition results and compared with ANN algorithms. Then, through some experiments, we presented the optimal architecture based on the results. Selecting the frame length determines only the input dimension of our method. The second challenge is to find an optimal architecture for the CNNs. Therefore, firstly, we defined the input and the output structure of the network.

## 3. Experiment Environment Setup

In order to develop a recognition system for the diagnosis of skin cancer, we should give specific answers for the following set of questions; this will give more grants for developing a successful system.

1. Does the real-time standard set used to examine the selected feature recognition system scores the highest ranking using the information methods?
2. Do the advanced artificial intelligence algorithms like CNNs have the capability to obtain the highest accuracy for detection the skin cancer?
3. Why should we compare the traditional machine learning algorithm results like ANNs and the deep learning CNNs used in detecting skin cancer?

The article "Developing a Recognition System for Diagnosing Melanoma Skin Lesions Using Artificial Intelligence Algorithms" was published in 2021. Journal: Comput Math Methods Med.

In order to give answers to the above questions, real-time stranded datasets were used. The ANN and CNN classification algorithms were applied to detect skin diseases. The implementation of this research has been done using Matlab 2020 programming. The experiments were conducted on the system with I7 Processor and 8 GB RAM to process all system tasks. The evaluation metrics were used to evaluate the proposed system. The classification results of ANN and CNN Algorithms are presented. The experimental results of the recognition system were tested and evaluated by employing the evaluative metrics: accuracy, sensitivity, specificity, precision, recall, and F1 score. The developing system was applied to diagnosis the skin cancer. The detailed description of the experiment results of the proposed system is presented in the following subsection.

### 3.1. Evaluation Metrics

In order to evaluate and measure the effectiveness of the recognition system, the performance measurement metrics like accuracy, sensitivity, specificity, precision, recall, and F1 score were employed. The equations are defined as below:

(21) $$\begin{array}{c} \text{Accuracy}=\frac{\text{TP}+\text{TN}}{\text{FP}+\text{FN}+\text{TP}+\text{TN}},\\ \text{Specificity}=\frac{\text{TN}}{\text{TN}+\text{FP}}\times 100\%\text{Specifity}=\frac{\text{TN}}{\text{TN}+\text{FP}}\times 100\%\\ \text{Sensitivity}=\frac{\text{TP}}{\text{TP}+\text{FN}}\times 100\%\text{Sensivity}=\frac{\text{TP}}{\text{TP}+\text{FN}}\times 100\%,\\ \text{Precision}=\frac{\text{TP}}{\text{TP}+\text{FP}}\times 100\%\text{Sensivity}=\frac{\text{TP}}{\text{TP}+\text{FN}}\times 100\%,\\ \text{Recall}=\frac{\text{TP}}{\text{TP}+\text{FN}}\times 100\%\text{Sensivity}=\frac{\text{TP}}{\text{TP}+\text{FN}}\times 100\%,\\ \text{F}1\text{ score}=2*\frac{\text{precision}*\text{Recall}}{\text{precision}*\text{Recall}}\times 100\%\text{Sensivity}=\frac{\text{TP}}{\text{TP}+\text{FN}}\times 100\%, \end{array}$$

where TP is true positive, FP is false positive, TN is true negative, and FN is false negative.

### 3.2. Splitting of Datasets

Table 3 provides a description setup of the skin disease datasets used in these experiments.

### 3.3. Experiment Results of the Artificial Neural Network (ANNs) Algorithm

In this section, the results of the ANN algorithm to diagnose skin cancer are presented. The datasets were divided into 80% training and 20% testing. The ANN algorithm was used as PH^2^ database to detect the skin diseases, whereas the PH2 dataset has three diseases, namely, common nevi, benign, and melanoma, whereas the ISIC 2018 has seven classes. We created a neural network with 10 hidden layers, 216 inputs, and 3 outputs.  Figure 14 shows the framework of the ANN model for PH2 and ISIC 2018 datasets to diagnose the skin diseases. In PH2 dataset, 27 epochs are considered for the training process. The confusion matrix of the ANN model of the PH2 dataset is displayed in Figure 15, whereas Figure 16 shows the confusion matrix of ANNs for the ISIC 2018 dataset. The confusion matrix consists of four training, validation, testing, and all data. Three epochs were achieved in the training process to obtained good performance, with time elapsed 3 min. The actual class is represented in the rows, and the predicted class is represented in the columns. The correct classification class represents in the trig diagram of the confusion matrix. The last cell rows display the accuracy of the model. By analyzing this result of the ANN algorithm, it is noted that that neural network with 10 hidden layers is more appropriate for distinguishing the malign lesion from the benign one.

The article "Developing a Recognition System for Diagnosing Melanoma Skin Lesions Using Artificial Intelligence Algorithms" was published in 2021. Journal: Comput Math Methods Med.

Table 4 summarizes the results of the ANNs to detect skin diseases. It is noted that the performance of the ANN model with ISIC 2018 dataset is very superior compared with PH2, but overall, the ANN model is more appropriate to diagnosis the skin diseases. It is noted that the ANNs with ISIC 2018 dataset attained the highest accuracy, (98.35%).

The performance plot is used to identify the mean square error in the network in order to diagnose skin diseases. It is useful to test the proposed. The performance of the ANN model is displayed in Figure 17. The best validation of the ANN model was 0.018149 at epoch 27 with PH2 dataset. In this case, ISIC 2018 best validation of the ANN model is 0.037798 at epoch 36. The performance of the ANN model means the square error rapidly decreases as it learns. The blue line indicates the training process, and a green line represents the validation error. The red line represents the error of testing the training. Additionally, when the number of epochs in the system increases, a smaller error in the training data will be obtained. When the validation error stops decreasing, the training also stops.

Figure 18 displays the gradient value of the training process at each iteration. The gradient value of the ANN-model-diagnosed skin diseases from the PH2 dataset is 0.018149 at epoch 33. The gradient value of the ANN model in ISIC 2018 is 0.0058777 at epoch 42. The performance validation check = 6 at epoch is presented.

The receiver operating characteristic (ROC) displays the simulation results of the ANN model to diagnose skin diseases.  Figure 19 shows the receiver operating characteristic (ROC) to measure validation of the ANN model using two real standard datasets. The graphic representation of testing, training, and validation of the system is presented. The last graph shows the overall ROC of the system.

The article "Developing a Recognition System for Diagnosing Melanoma Skin Lesions Using Artificial Intelligence Algorithms" was published in 2021. Journal: Comput Math Methods Med.

### 3.4. Experiment Results of the Deep Learning Algorithm

This section presents the simulation results of two CNNs (AlexNet and ResNet50) for detecting skin diseases. The dataset was divided into 80% training and 20% testing. In order to obtain powerful results, the input size should be fixed. In this research, the input size is a 244 × 244 × 3 matrix. The output shape in this present research is the softmax function, with three classes for the PH and seven classes for the ISIC 2018 datasets. The softmax layer is used as an output to recognize skin diseases from both datasets. The performance of the CNNs (AlexNet and ResNet50) depends on the CNN parameters such as filter size, hidden layer, and the number of filters used in the convolutional layer. In the AlexNet transfer model, 34 layers and 10 epochs were utilized. The PH 2 and ISIC 2018 datasets were used with different outputs to test the AlexNet and ResNet50. The input data of PH2 120 images and ISIC 2018 is 840 images. In the ResNet50 transfer model, 174 hidden layer and minibatch size of one, while the weight learning rate factor and the bias learning rate factor were set to 20; the epoch's values are 10. The number of feature maps is usually equal to the number of filters used. Pooling size also affects the accuracy of the network result, and when used, it fully connects the number of nodes used at this layer. The number of convolutional layers has a significant effect on the result. We cascaded the convolutional layers together to build our classifier system. Each convolutional network consists of convolution, nonlinearity, pooling layers.

The (AlexNet and ResNet50) transfer learning model has applied as individual classifiers for skin diseases detection. From each database, 80% of the images were used for training, and 20% of the images were used for validation (in both PH 2 and ISIC 2018).  Table 5 shows the results of the AlexNet model, and the results of the ResNet50 model are presented in Table 6. It is observed that the results of ResNet50 are better than AlexNet. The results of ResNet50 have a higher accuracy which indicates that it plays a leading role in the proposed model.  Figure 20 shows the confusion Metrix of AlexNet for detecting skin diseases using PH2 and ISIC 2018.  Figure 21 shows the confusion matrix of ResNet50 for both datasets and presented several sample validation images. For each of them, we presented the predicted labels and the predicted probabilities of the images having those labels.

The article "Developing a Recognition System for Diagnosing Melanoma Skin Lesions Using Artificial Intelligence Algorithms" was published in 2021. Journal: Comput Math Methods Med.

Figure 22 displays the ROC curve for the AUC stand metric of the AlexNet model for both datasets. The ROC curve for AUC stand metric of ResNet50 is shown in Figure 23. The graphical representation demonstrates the successful classification; the false positive rate is very low. The blue line shows the detection rate; it is noted that the detection rate is very high for recognizing skin diseases. The figure indicates that the performance of the AlexNet and Resnet-50 models is good multiclass ROC curve, and it attains a statistically significant AUC value of 94.05% of ResNet50 with ISIC datasets.

## 4. Discussion

In this research work, developing the proposed system using artificial intelligence to detect skin diseases is presented. Two real standard datasets were employed for evaluating the proposed system. The datasets were split into 80% for training state and 20% for the testing state. The proposed system was developed using Matlab.

Initially, we developed a system based on the features obtained from the extraction methods. The hybrid feature extraction, based on LBP and GLCM, was implemented to extract significant features. The hybrid feature extraction methods extruded 216 significant features. These features were processed using the ANN algorithm in order to detect skin diseases. In the ANNs model, we considered 10 hidden layers regarding 216 input and seven output features for ISIC 2018 and 3 for PH2 datasets. Notably, the ANNs achieved the highest accuracy for ISIC datasets: accuracy = %. In the second model, the deep learning algorithm was proposed. Two transfer learnings, namely, AlexNet and ResNet50, were considered for skin disease detection. The results of ResNet50 are better for both datasets.

Overall, it was observed that the ANN model achieved the highest accuracy compared with using the CNN algorithm. In the case of the ANN model, we preprocessed all images to remove the hair from images; this helped increase the accuracy of the proposed model. The developed diagnosis system's most prominent challenges are due to the similarity of skin disease features. Another issue is the quality of the images, which look like dermatologist-drawn makings into the lesion. However, the developing system has the ability to detect skin diseases with accuracy (98.35%). Comparative classification results between the proposed model and the existing one are displayed in Table 7.

The proposed methodology's empirical results are highly accurate (98%) using the ANN algorithm based on ISIC 2018, and the ANN model based on PH2 data achieved an accuracy of 97.50%. Additionally, the CNN transfer learning model attained satisfactory results compared with existing models. Finally, we believe that the proposed system has the ability to diagnose skin diseases.

The article "Developing a Recognition System for Diagnosing Melanoma Skin Lesions Using Artificial Intelligence Algorithms" was published in 2021. Journal: Comput Math Methods Med.

## 5. Conclusion

Nowadays, it is essential to focus more attention toward the early detection of skin diseases such as melanoma before they spread to other parts of the body. In this research, we developed a skin diagnosis system based on AI algorithms. The proposed methodology was evaluated and tested using statistical analysis methods. The following conclusions can be drawn from the use of advanced AI for the classification of skin diseases:

- Two real standard datasets were used to test and evaluate the diagnostic system
- ANN algorithms based on features that were extracted from skin lesions using hybrid feature extraction methods were implemented. The developed database contains 216 significant features that can be considered important for skin disease diagnosis
- CNN transfer learning, AlexNet and ResNet50, was applied to classify the skin diseases
- Comparisons between the ANN-based on features and CNN algorithm are presented. It is noted that the ANN algorithm achieved the highest accuracy
- We tested the proposed system by detecting skin diseases
- Comparative classification results between the proposed system and existing system are presented. Overall, the proposed system achieved good accuracy and is more satisfactory

## Figures and Tables

**Figure 1:** Malignant melanoma cancer images.

**Figure 2:** Formwork of the proposed system.

**Figure 3:** Simple images extracted from the PH2 database.

**Figure 4:** Simple images extracted from the ISIC 2018 database.

**Figure 5:** The steps of skin disease detection using the feature-based method.

**Figure 6:** Segmentation PH2 images using the active contour method: (a) atypical nevi, (b) common nevus, and (c) melanoma.

**Figure 7:** Segmentation ISIC 2018 images using the active contour method: (a) melanocytic nevi (nv), (b) melanoma (mel), (c) benign keratosis lesions (bkl), (d) basal cell carcinoma (bcc), (e) actinic keratoses (akiec), and (f) vascular (vasc) 100.

**Figure 8:** LBP neighborhood pixels.

**Figure 9:** Architecture of the ANN algorithm: (a) architecture of ANNs using PH2 and (b) architecture of ANNs using ISIC 2018.

**Figure 10:** Working of CNN with many convolutional layers.

**Figure 11:** ReLU function.

**Figure 12:** Fully connected layer: (a) ISIC 2018 dataset and (b) PH2 dataset.

**Figure 13:** AlexNet introduced by Krizhevsky 2014 [40].

**Figure 14:** Framework of the FFNN model: (a) PH2 dataset and (b) ISIC 2018.

**Figure 15:** Confusion matrices in case of the PH2database.

The article "Developing a Recognition System for Diagnosing Melanoma Skin Lesions Using Artificial Intelligence Algorithms" was published in 2021. Journal: Comput Math Methods Med.

**Figure 16:** Confusion matrices in case of the ISIC 2018 database.

**Figure 17:** Performance plot of the training process: (a) PH2 dataset and (b) ISIC 2018.

**Figure 18:** Displays the gradient value of the training process: (a) PH2 dataset and (b) ISIC 2018.

**Figure 19:** Receiver operating characteristic (ROC): (a) PH2 dataset and (b) ISIC 2018.

**Figure 20:** Confusion matrices AlexNet in case of (a) PH2 and (b) ISIC 2018.

**Figure 21:** Confusion matrices ResNet in case of (a) PH2 and (b) ISIC 2018.

**Figure 22:** ROC curve of the AlexNet model: (a) PH2 and (b) ISIC 2018.

**Figure 23:** ROC curve of the ResNet-50 model: (a) PH2 and (b) ISIC 2018.

**Table 1:** Significant parameters of the AlexNet model.

Layer No.	Elements	Parameters	Values
1	Convolutional filter	Input channels	3
		Size	11 × 11
		Stride	4 × 4
		Padding	3 × 3 × 3
	Max-pooling	Pool size	3 × 3
		Padding	1 × 1 × 1 × 1

4	Fully connected	Input to layer	192 × 2 × 2
		Output from layer	177

5	SoftMax	Output units	7 and 3

**Table 2:** Significant parameters of the ResNet50 model.

Layer No.	Elements	Parameters	Values
1	Convolutional filter	Input channels	3
		Size	7 × 7
		Stride	2 × 2
		Padding	3 × 3 × 3
	Max-pooling	Pool size	3 × 3
		Padding	1 × 1 × 1 × 1

4	Fully connected	Input to layer	192 × 2 × 2
		Output from layer	177

5	SoftMax	Output units	7 and 3

**Table 3:** Distribution and splitting of the used datasets.

Dataset name	Total of samples	Training set (70%)	Testing set (30%)	Total of classes
ISIC 2018	840	672	168	7 classes
HP2	120	96	24	3 classes

**Table 4:** Results of the ANN model.

Datasets	Accuracy (%)	Sensitivity (%)	Specificity (%)	Precision (%)	*F*-score (%)
PH2	97.50	98.30	96.72	96.66	97.47
ISIC 2018	98.35	99.41	97.33	97.27	97.47

**Table 5:** Results of the AlexNet model.

Datasets	Accuracy (%)	Sensitivity (%)	Specificity (%)	Precision (%)	*F*-score (%)
PH2	91.67	100	88.89	75.0	85.71
ISIC 2018	88.10	75.00	88.41	80.50	80.84

**Table 6:** Results of the ResNet50 model.

Models	Accuracy (%)	Sensitivity (%)	Specificity (%)	Precision (%)	*F*-score (%)
PH2	91.67	87.50	93.50	87.50	87.50
ISIC 2018	94.05	97.50	92.97	81.25	88.64

**Table 7:** Comparsion results using accuracy metric.

References	Methods	Accuracy	Observation	Datasets	Size of datasets
[43]	Deep learning, SVM	93.1%	Classification	ISIC	2146
[44]	CNNs	85.5%	Classification	ISIC 2017	1300
[45]	CNN-feature-based	81%	Classification	PH2	50
[46]	CNNs	91.2%	Classification	ISIC 2017	2000
Proposed model (ANNs)		97.50 98.35	Classification	PH2 ISIC 2018	120 840
Proposed model (CNNs)		91.67 94.05	Classification	PH2 ISIC 2018	120 840

## Data Availability

The researchers can collect data from this link: https://www.fc.up.pt/addi/ph2%20database.htmlhttps://dataverse.harvard.edu/dataset.xhtml?persistentId=doi:10.7910/DVN/DBW86T.
